The article "Effect of Clinical Nursing Pathway Intervention Based on Evidence-Based Medicine on Venous Thrombosis in Long-Term Bedridden Patients" was published in 2022. Journal: J Healthc Eng.

# Effect of Clinical Nursing Pathway Intervention Based on Evidence-Based Medicine on Venous Thrombosis in Long-Term Bedridden Patients

**DOI:** 10.1155/2022/5120569

**Published:** 2022-03-14

**Authors:** Jing Chen, Yanli Wen, Lin Jin, Junwei Peng, Jin Ji

**Affiliations:** ^1^Department of Cardiothoracic and Vascular Surgery, Suizhou Hospital, Hubei University of Medicine, Suizhou, Hubei Province, China; ^2^Department of Neurology, Suizhou Hospital, Hubei University of Medicine, Suizhou, Hubei Province, China; ^3^Department of Critical Care Medicine, Zengdu Hospital, Suizhou, Hubei Province, China; ^4^Department of Nursing, Suizhou Hospital, Hubei University of Medicine, Suizhou, Hubei Province, China

## Abstract

**Background:**

Venous thrombosis is a type of medical condition that establishes as deep vein thrombosis of the limb or pulmonary embolism. This disease arises as a result of interrelating hereditary, ecological, and interactive risk aspects. Clinical nursing pathways also known as critical pathways are pathways that guide nurses when developing a patient's care plan. However, the effect of nursing intervention on venous thrombosis in long-term bedridden patients from the perspective of evidence-based medicine had not been reported.

**Methods:**

A total of 170 patients hospitalized in the hospital from January 2021 to October 2021 were selected, and the bed time was more than 2 weeks. The patients were randomly divided into the control group and observation group. 85 cases in the control group received routine nursing in cardiology, and 85 cases in the observation group received clinical nursing pathway. Venous thrombosis, lower limb pain, swelling, D-dimer level, hemodynamic parameters, and nursing satisfaction were compared in two groups.

**Results:**

The incidence of deep venous thrombosis in the observation group was 8.2%, lower than 24.7% in the control group (*P* < 0.05). The incidence of lower limb pain and elevated D-dimer in the observation group was lower than that in the control group (*P* < 0.05). The improvement of hemodynamic parameters such as SBP, DBP, CBV, PR, CI, and CO in the study group was better than that in the control group (*P* < 0.05). The satisfaction of the observation group was 90.58%, which was higher than that of the control group (82.35%) (*P* < 0.05).

**Conclusion:**

Clinical nursing pathway can improve patients' nursing efficiency, improve the treatment effect, shorten hospital stay, and improve nursing satisfaction.

## 1. Introduction

Venous thromboembolism included deep venous thrombosis and pulmonary thromboembolism [1]. Deep venous thrombosis referred to abnormal blood coagulation in deep veins, resulting in venous reflux disorder, resulting in deep venous insufficiency [2]. The main manifestations were lower limb pain, swelling, and movement disorder. Thrombus shedding could also lead to pulmonary embolism and life-threatening. Venous thromboembolism usually occurred in the deep veins of the leg and thigh [2]. According to the reported statistics, the incidence of venous thrombosis in long-term bedridden patients was as high as 31%, which is significantly higher than that in nonbedridden patients [3]. The main causes in long-term bedridden patients included cerebrovascular diseases, bone and joint diseases, tumors and organ failure, pregnant women after cesarean section, and old age, which were often combined with the first three causes. Aging population was gradually increasing, and elderly long-term bedridden patients were the high-incidence population of deep venous thrombosis [4]. Deep venous thrombosis of lower limbs is a common complication of the elderly in bed for a long time and limb fixation during and after operation, which often leads to slow venous blood flow, hypercoagulable blood state, and venous wall injury. Certain nursing intervention can improve the hypercoagulable blood state of the body, accelerate the blood flow rate, and promote the recovery and improvement of vascular perfusion of lower limbs local blood circulation to prevent the occurrence of lower extremity deep venous thrombosis. At present, the treatment of venous thrombosis is mainly drug anticoagulant and thrombolytic therapy. Although thrombolytic and anticoagulant therapy is performed, some patients would develop deep venous thrombosis syndrome, which seriously affected the quality of life of patients. Therefore, prevention is greater than treatment for venous thromboembolism [5]. With the development of the times, traditional nursing based on experience was changing to modern nursing based on science. There were evidences to follow, which could provide more comprehensive and scientific guidance for nursing work [6]. Clinical nursing pathway is an interdisciplinary, comprehensive, and deepening overall clinical nursing work mode. It is a method to promote treatment organization and disease management under the guidance of evidence-based medical evidence and guidelines. It could standardize medical behavior, reduce nursing cost waste, and improve patients' quality of life. Previous studies had found that evidence-based nursing could improve the clinical cure rate of patients with malignant tumors complicated with lower extremity venous thrombosis and significantly improve the quality of life of patients [7]. The use of clinical nursing pathway after femoral fracture surgery could effectively prevent the occurrence of deep venous thrombosis and improve the coagulation function of patients [8]. Clinical nursing pathway intervention could effectively reduce the incidence of lower extremity venous thrombosis after total hysterectomy [9]. It could be seen that the clinical nursing pathway intervention model had been widely carried out in many clinical disciplines and had played an important role in the prevention and treatment of venous thrombosis. Therefore, this study was based on evidence-based nursing, query data, formulate practical clinical nursing path measures, and explore its impact and application value on the prevention of venous thrombosis in long-term bedridden patients.

## 2. Methods

### 2.1. Clinical Information

A total of 170 patients hospitalized in the hospital from January 2021 to October 2021 were selected, and the bed time was more than 2 weeks. They were randomly divided into the observation group and control group, with 85 cases in each group. Underlying diseases include stroke, coronary heart disease, coronary heart disease, diabetes, hypertension, fractures, and no venous thromboembolism. Patients and their families voluntarily joined and signed the consent form, requiring them to cooperate with nursing work. In the observation group (37 males and 48 females), the age ranged from 57 to 83 years, with an average of (70.9 ± 7.5) years. In the control group (41 males and 44 females), the age ranged from 55 to 79 years, with an average of (69.8 ± 7.1) years. The general data of the two groups were statistically processed, and the difference was not statistically significant (*P* > 0.05).

### 2.2. Nursing Intervention Measures

The control group was treated with routine prevention and intervention methods, including the use of anticoagulants, raising the lower limbs and massage, wearing elastic socks, and routine health education.

In the observation group, evidence-based medicine was used to intervene the clinical pathway of long-term bedridden patients. A clinical pathway nursing team with head nurse as the team leader and responsible doctors and nurses as members was established to find the literature and data and summarize the relevant factors and the latest preventive measures of venous thrombosis according to the problems and hidden dangers in previous routine nursing. According to the actual situation of the department and the individual differences of long-term bedridden patients, combined with the lower extremity venous thrombosis score scale, the relationship between many related factors of lower extremity venous thrombosis and patients was evaluated, and a scientific clinical nursing path to intervene bedridden patients was formulated. The team members should be trained accordingly, including knowledge of venous thrombosis, characteristics of the clinical nursing path, and implementation process so as to improve the nursing skills of the team members and ensure the effective development of nursing work.

1. Patient risk assessment and health education at admission: the medical staff used the venous thrombosis risk assessment form of our hospital and combined with the patient's examination results to evaluate the risk of venous thrombosis and recorded it in the patient's cases so as to provide reference for later treatment and nursing. When the condition changes, it needed to be reassessed. Mastering the patient's educational level and understanding of venous thrombosis is the basis of personalized health education. Combined with health manuals and videos, patients' understanding of venous thrombosis and its harm was deepened and made them to preliminarily grasp their own risk of venous thrombosis, which can increase patients' compliance in the later stage. The rewritten sentence is as follows: Due to long-term bed rest, patients are prone to have negative emotions, so it is necessary to communicate closely with patients and their families, and choose personalized health education to relieve patients' negative emotions. Nurses should understand the living habits and eating habits of patients. Patients were guided to drink more water and follow the doctor's advice to ensure that they were supplemented with enough liquid to prevent blood concentration. Eating vegetables and fruits rich in fiber and ensuring low sugar, low salt, low fat, and high vitamins reduce constipation and prevent the increase of abdominal pressure from affecting the venous reflux of lower limbs [10]. The patient's bad life behaviors, such as drinking and smoking, were corrected.
2. Lower limb functional exercises: after admission, patients were supervised and assisted with lower limb functional exercise to avoid lower limb venous thrombosis. After admission, appropriate elastic socks were selected to prevent lower limb blood stasis, but it should be noted that patients with ischemic stroke should avoid using elastic socks [11, 12]. Patients were given intermittent lower limb compression twice a day to increase lower limb muscle movement. However, it should be noted that the contraindications of intermittent pressure inflation pump include leg diseases, such as open wound, dermatitis, gangrene, severe edema, lower limb venous congestion, severe peripheral vascular diseases, postoperative venous ligation or transplantation, heart failure, unclear consciousness, and swelling or other symptoms of existing venous thrombosis. Attention was paid to prevent cross infection during use [13, 14]. At the same time, the patient's family members were guided to perform passive movements of the patient's lower limbs, including leg elevation, knee flexion, and joint activities, for 20–30 min each time. To increase gastrocnemius muscle compression and ankle pump movement to assist patients with internal and external somersault, extension and flexion of the ankle for more than 5 min were performed [15]. To guide the patient to raise the affected limb, the patient was guided to hold the sole of the foot with his left hand under the knee and his right hand and carry out activities such as internal and external rotation and abduction and adduction for more than 12 min. The range of activities could be gradually increased, but the strength was controlled within the patient's tolerance [16].
3. Prevention of the occurrence of lower extremity venous injury: during intravenous infusion, upper limb venipuncture can be chosen and healthy limb puncture can be selected for patients with hemiplegia [17]. For patients with long-term infusion, intravenous indwelling needle could be used. It was recommended to use indwelling venous catheter in the upper limb or under the clavicle to reduce the number of puncture [18]. The nursing was strengthened, damage to the blood vessel wall was prevented, and the incidence of thrombosis was reduced. The use of precision infusion set during infusion could avoid the entry of particles in the vein. At the same time, the drug dose could be adjusted in time according to the needs of the patient's condition so as to reduce drug residue, reduce the stimulation to blood vessels, and avoid phlebitis.
4. Condition observation and patrol inspection: the affected limb was checked every day; the skin, pulse, heart rate, and dorsal foot artery around the affected limb were closely monitored; adverse symptoms such as fever, pain, and swelling were observed for occurrence; and the peripheral diameter of the affected limb was measured and recorded. As the patient was bedridden for a long time, skin care was also very important. Nurses needed to regularly supervise the family members to pat the patient's back, wipe the bath, massage, and turn over so as to avoid skin complications [19]. In case of any abnormality, communication with the doctor in time and dealing with it in time have to be carried out.

### 2.3. Observation Indicators

After evidence-based nursing intervention, the clinical manifestations, symptoms, signs, and laboratory examination results of long-term bedridden patients were analyzed. The results of venous thrombosis, lower limb pain, swelling, D-dimer level, hemodynamic parameters, and nursing satisfaction were compared between the two groups.

### 2.4. Statistical Methods

The SPSS 25.0 statistical software was used to measure the data, and independent sample *t*-test was used, including lower limb pain, swelling, D-dimer level, and hemodynamic parameters. Counting the data, using the *χ*^2^ test, including venous thrombosis and nursing satisfaction, was performed. The difference was significant or statistically significant (*P* < 0.05).

## 3. Results

Table 1 shows a comparison of the incidence of complications and venous thrombosis. In the control group, 17 patients had lower limb pain, 8 patients had lower limb swelling, 27 patients had positive elevation of D-dimer, and 21 patients had venous thrombosis. In the observation group, 5 patients had lower limb pain, 4 patients had lower limb swelling, and 9 patients had positive elevation of D-dimer. After further examination, 7 patients were diagnosed with venous thrombosis, and the other patients had no thrombosis. The incidence of venous thrombosis in the observation group was 8.2%. The incidence of venous thrombosis in the control group was 24.7%. There was significant difference in the incidence of venous thrombosis between the two groups (*χ*^2^ = 8.380, *P* = 0.004), as shown in Table 1.

Table 2 shows the comparison of hemodynamic indexes in patients. The improvement of hemodynamic parameters such as SBP, DBP, CBV, PR, CI, and CO in the observation group was better than that in the control group (*P* < 0.05), as shown in Table 2.

Table 3 shows the nursing satisfaction rate. Comparison of nursing satisfaction between the two groups is shown in Table 3. The nursing satisfaction of the observation group was 90.58%, which was significantly better than that of in the control group (82.35%) (*P* < 0.05).

## 4. Discussion

Venous thrombosis was one of the common complications of long-term bedridden patients. Its occurrence and development were inseparable from basic diseases and old age [20]. The literature showed that history of thrombosis, hypertension, hyperlipidemia, and diabetes would cause the body to be in a hypercoagulable state. Reduced body activity could cause blood stasis, aggravate hypercoagulability, slow venous blood flow, and increase the risk of thrombosis [21]. The blood vessels of elderly patients could have degenerative lesions, reduced vascular elasticity, rough intima, and easy to be damaged. The latest domestic research found that the clinical nursing pathway could effectively improve the probability of lower extremity deep venous thrombosis and joint dislocation after hip arthroplasty and improve patients' nursing satisfaction and treatment compliance [22]. It could promote the early postoperative rehabilitation of elderly patients with femoral neck fracture and reduce the incidence of deep venous thrombosis [23]. The clinical nursing pathway had also achieved good results in the nursing of patients with intracerebral hemorrhage [24]. Evidence based nursing was based on science, aiming at the detailed problems found in the process of nursing practice, making nursing decisions, and guiding clinical nursing work by querying and collecting materials [25]. Using the concept of evidence-based medicine in nursing work could better expand the thinking of nurses so as to carry out nursing work more scientifically and reasonably. The nursing practice project of preventing venous thrombosis based on evidence-based medicine could improve nurses' cognition of deep venous thromboembolism, actively evaluate the risk of deep venous thrombosis, standardize the management process, and avoid the waste of clinical nursing resources [26]. Making the nursing path plan according to the patient's condition and evidence-based medicine nursing method could reduce the occurrence of clinical adverse events and shorten the rehabilitation time of patients. Compared with the guidelines, the nursing pathway was a diagnosis and treatment process for specific diseases [27]. It paid attention to the synergy between various specialties in the treatment process and is more time-effective.

Before or during thrombosis, it was often accompanied by sensory abnormalities such as limb swelling and numbness as well as pain leading to claudication. D-dimer quantitative examination was very sensitive in the diagnosis of lower extremity deep venous thrombosis. Positive could not predict specific diseases, but it has a negative exclusion diagnostic value, which was very useful in the diagnosis of suspected deep venous thrombosis [28]. Therefore, we choose these indicators to assist in the evaluation of the nursing effect. Our results showed that the incidence of venous thrombosis was 8.2% in the observation group and 24.7% in the control group, indicating that the incidence of thrombosis was significantly reduced by using the clinical nursing pathway intervention model for long-term bedridden patients. In the control group, 17 patients had lower limb pain, 8 patients had lower limb swelling, and 27 patients had elevated D-dimer. In the observation group, 5 patients had lower limb pain, 4 patients had lower limb swelling, and 9 patients had positive elevation of D-dimer. The incidence of adverse events in the control group was 61.2%, which was higher than 21.2% in the observation group. The conclusion showed that the clinical nursing path based on evidence-based medicine plays a better role in preventing venous thrombosis and adverse complications in long-term bedridden patients compared with the conventional nursing model [29]. Compared with the conventional nursing mode, personalized health education for patients could better improve the compliance of patients. Supervising the regular lower limb movement of patients could prevent patients and their families from taking chances and being lazy and could effectively prevent lower limb venous thrombosis [30]. Our results once again confirmed that the clinical nursing pathway intervention model based on evidence-based medicine is worthy of wide promotion in clinic. The study results showed that the nursing satisfaction of the observation group was 90.58%, which was significantly better than that of the control group (82.35%). At the same time, the improvement of hemodynamic parameters such as SBP, DBP, CBV, PR, CI, and CO in the observation group was better than that in the control group. In the process of nursing patients, we should assist patients in limb movement, which could effectively improve the blood flow velocity of patients and prevent the formation of venous thrombosis [31]. At the same time, attention to the limb pain and swelling of patients has to be paid. If abnormalities were found, diagnosis should be performed as soon as possible and measures for intervention should be carried out.

## 5. Conclusion

In conclusion, the implementation of nursing pathway intervention based on evidence-based medicine had effectively reduced the incidence of lower extremity venous thrombosis in long-term bedridden patients. Clinical nursing pathway can improve patients' nursing efficiency, improve the treatment effect, shorten hospital stay, and improve nursing satisfaction. At the same time, our research also confirmed the accuracy, scientificity, and practicality of evidence-based nursing.

## Figures and Tables

**Table 1:** Comparison of the incidence of complications and venous thrombosis (n, %).

Groups	N	Venous thrombosis	Pain	Swelling	D-dimer elevation
Control group	85	21 (24.7%)	17 (20%)	8 (9.4%)	27 (31.8%)
Observation group	85	7 (8.2%)	5 (5.9%)	4 (4.7%)	9 (10.6%)
*χ* ^2^		8.380	7.518	1.435	11.418
*P* value		0.004	0.006	0.231	0.001

**Table 2:** Comparison of hemodynamic indexes in patients (n, %).

Groups	*N*	SBP (mmHg)	DBP (mmHg)	CBV (L)	PR (mmHg/l.min)	CI (L/min.m^2^)	CO (L/min)
Control group	85	124.14 ± 16.8	70.61 ± 7.2	0.83 ± 0.12	18.14 ± 2.36	2.02 ± 0.26	3.41 ± 0.56
Observation group	85	133.11 ± 16.7	73.63 ± 7.8	1.14 ± 0.13	23.31 ± 2.62	2.24 ± 0.36	5.71 ± 0.86
*t*		12.254	20.271	24.268	17.479	15.452	18.369
*P* value		0.014	0.008	0.006	0.007	0.011	0.009

**Table 3:** Nursing satisfaction rate (n, %).

Groups	*N*	Satisfied	Basically satisfied	Dissatisfied	Overall nursing satisfaction
Control group	85	35 (41.18%)	35 (41.18%)	15 (17.65%)	70 (82.35%)
Observation group	85	37 (43.53%)	40 (47.06%)	4 (4.7%)	77 (90.58%)
*χ* ^2^					12.629
*P* value					0.001

## Data Availability

The simulation experiment data used to support the findings of this study are available from the corresponding author upon request.
